The article "Internet-Based Approaches to Designing an Online Fitness Platform" was retracted in 2023. Reasons: unreliable results or conclusions; concerns about the data; concerns about the peer review; concerns about the citations.

# Internet-Based Approaches to Designing an Online Fitness Platform

**DOI:** 10.1155/2022/9113569

**Published:** 2022-01-25

**Authors:** Bo Liu

**Affiliations:** Chengde Medical University, Chengde 067000, Hebei, China

## Abstract

In recent years, national fitness has become a hot topic. How to take healthy and effective exercise on a daily basis is an urgent problem to be tackled. Web-based platforms are accessible through cellphones, which include fitness records, teaching videos, and result feedback. These three aspects assist users in completing their initial evaluation, which further contributes to health improvement. Additionally, enhancement in the well-being of individuals is carried through video recommendations. In order to proceed fitness related videos suggestions, this platform uses a collaborative filtering algorithm, which is based on videos recommendation. To receive suggestions, this methodology acquires five queries to be completely addressed at the preliminary stage. This initial assessment is commonly known as a cold-start evaluation strategy. Furthermore, popularity punishment measures are incorporated to enhance productivity. Finally, this platform offers an online-based approach for the inspection, assessment of the national fitness, and orientation for the future improvement of the fitness database.

## 1. Introduction

With the advent of sophisticated technological accessories, lifestyle is changed in many ways. The convenient accessibility of these portable devices, especially cellphones, serves humanity in numerous walks of life. Although the living standards of individuals have improved, they bring several challenges to society. On the other side of such innovations, reduction in face-to-face interaction occurs, which leads to several health and psychological issues [1]. Eventually, body fitness is no longer the priority of a specific age-based group. In the end, figure is no longer the priority of a certain age group, but it needs to be paid attention to in the whole society, regardless of age and gender. Since 2009, the national fitness day has been celebrated annually. National fitness has become an essential part of daily life. The original purpose of national fitness is to enhance the physiques of teenagers. Especially, the increasing rate of diseases amongst older encourages them to join this platform. Besides old-age people, the young generation is interested in connecting it due to enormous benefits in sports. According to Shanghai 2017 census, public fitness places continue to escalate. Consequently, sporting areas continue to increase to 3.143,000 square meters. Public fitness places expand, and per capita reaches 1.96 square meters. Therefore, searching for healthy and effective exercise became a global challenge [2–4].

The article "Internet-Based Approaches to Designing an Online Fitness Platform" was retracted in 2023. Reasons: unreliable results or conclusions; concerns about the data; concerns about the peer review; concerns about the citations.

The ultimate goal of nationwide fitness centers can improve the citizen's health through regular exercise. Lack of exercise expertise sometimes results in severe sort of injuries; that is why appropriate guidelines are essential to boost one's performance in sports. When exercise time is appropriate and the method is suitable, then citizen enjoys flexibility in games that effectively increase coordination. National fitness advocates citizens to participate in one or two types of activities on a daily basis and utilize different varieties of fitness approaches while playing. For most citizens, it is difficult to ensure daily access to professional movement guidance. Therefore, fitness activities have a significant impact on health as well body physique, which is often not worth the cost. In the process of attaining physical fitness, a single approach is not sufficient to achieve remarkable fitness results. Research depicts that best fitness is obtainable through two types of exercise in one session. To sum up, citizens' learning of fitness time and methods has become extremely important. The national fitness campaign calls for regular system testing for citizens. The physical fitness feedback data at different stages can effectively monitor the change of physical condition so as to facilitate timely adjustment of exercise mode [5–8].

Mobile Internet refers to the access to the Internet through wireless network technology, which can efficiently realize mobile Internet access. Therefore, the combination of national fitness with mobile Internet technology can provide users with fitness learning and other services in real time so as to facilitate users to use various available learning resources in the process of exercise. The national fitness online platform based on mobile Internet can provide users with three main services: correct learning of various fitness methods, recording of fitness activities, and recording of physical fitness [2, 3, 9]. The major contribution points of this research paper are given as follows:

- Designing an online-based platform for fitness
- Improvement in general exercise
- Easy approaches are utilized to make the public aware of online fitness platforms
- Assessment of public health on the national level

## 2. Literature Review

The old and traditional approaches to fitness have changed with the advent of the Internet. Exercise application decreases the expense of fitness where citizens achieve professional fitness information at their comfort zone by following lessons to enhance the corresponding exercise. The research study concluded that constructive trend develops through online national platform [2, 10]. Across the globe, countries pay huge attention to fitness at the former stage and improve their online application tends, which need to be advanced. In recent years, fitness applications in China have become common, while some high-quality fitness software emerged [19]. Besides Chinese innovations, other countries have developed their online platforms, such as the United States seven fitness O2O companies Fitstar, Fitmob, Runkeeper, Strava, Pact Fitness, MyFitnessPal, and Fitbit. These online applications provide individuals with effective fitness facilities through gathering personal data, growing social connections, and using psychological approaches [1]. Every platform has its own methods to access and collect personal health records. Fitstar offers teaching sessions and reservations by cooperating with nearby health care centers. Users of Fitmob request online colleagues to compete with others to work out [11]. Cash incentive is the function of Pact Fitness. Users join specific care centers through online and offline cooperations and get prizes or cash incentives by completing the proposed task. In case users are unable to complete the specific objective, users will be fined, which encourages them to increase exercise skills [9, 12]. However, in the Chinese market, there are some high-quality applications such as Keep, Gudong exercise, and weight loss king [13]. Gudong exercise offers social connections, and GPS (the global positioning system which is used to record and locate user's position) tracks the walking route and records the user's exercise performance. Weight loss king offers an inclusive slimming system for users, which analyzes body mass index. Various applications offer a wide range of lessons as video teaching resources, function of fitness trajectory, and social interaction [8, 14, 15].

The article "Internet-Based Approaches to Designing an Online Fitness Platform" was retracted in 2023. Reasons: unreliable results or conclusions; concerns about the data; concerns about the peer review; concerns about the citations.

### 2.1. The Overall Framework of the Online Platform

The framework of the online fitness platform is shown in Figure 1. Fitness users first acquire to log in to the application through a valid account and password. For first-time users, there are four types of questions to be addressed, such as gender, age, type of exercise, and location information. Each user should select at least 3 different varieties of exercise. Recommendations of videos and related tutorials are based on the users' exercise preferences [10, 16].

After successful log-in to the online interface, users are assisted with three modules, namely, punch module, teaching module, and recommended video module. The clocking module is used to record users' daily, weekly, monthly, and annual sports information. The teaching module provides users with a large number of high-quality fitness action videos. The users not only independently choose the types and quantity of videos to watch but also endorse fitness videos due to past history. For instance, a jogger might prefer the initial steps of yoga to calisthenics, while in recommendations, we should not be restricted to the accuracy of recommending video but also pay attention to the variety of recommended video, which must be sufficient to provide users with the possibility of trying other unexperienced sports. Finally, the feedback diagram of physical information can be viewed on the mobile Internet terminal by integrating various information of user [1, 4, 5, 7, 16].

With the improvement of living standards and the popularization of health concepts, individuals are paying more attention to their living conditions and health conditions, and various platforms have emerged as the times require. Individuals are connected through the platform and guided by data analysis. Therefore, spontaneous community association activities will become a trend where sports social organizations will become the main way for public sports participation [16].

### 2.2. Video Type Setting

The data were released in the 2017 national fitness development report of Shanghai; according to citizen priorities in selecting fitness methods, the most popular one is still walking as 19%. In addition, running 19%, dancing 12%, swimming 10%, badminton 10%, and other sports were selected as shown in Figure 2.

The number and type of teaching videos are selected according to specific situations of citizens in the actual process of exercise. There are many choices of brisk walking; therefore, resources allow a video library to set videos regarding the speed, time, and pace. On the other hand, there are numerous videos for dance as the demand for dance is much higher than other exercises. Hence, more categories are set under the option of dance, such as yoga, pas de deux, and aerobics [3, 11, 16].

To strengthen the proposed design of online sports facilities, various tools are utilized. Nowadays, the market for fitness is high as the population expands. Furthermore, the new technology fulfills the basic needs of society in terms of cultural and sports activities. Massive expansion in sports venue highlights its importance and urgent demand. The fitness priorities of people have evolved from shaping body shape to maintain a healthy body. At the present stage, large-scale commercial fitness clubs in cities are gradually increasing their health lectures, beauty and large-scale membership, and derivatives such as activities and catering services within the clubhouse. Therefore, China presents a comprehensive fitness club with cross industry. Chinese fitness companies are in the initial development stage, but still, there are huge opportunities for growth. With the advent of the latest technologies such as mobile Internet, online fitness applications changed human life [2, 3, 5, 17, 18].

The article "Internet-Based Approaches to Designing an Online Fitness Platform" was retracted in 2023. Reasons: unreliable results or conclusions; concerns about the data; concerns about the peer review; concerns about the citations.

### 2.3. The Primary Selection of Video Library

Based on the user's basic information, an effective filter must be formulated. Tags are divided into five main categories, as shown in Table 1. However, the videos' library can be preliminarily screened by current time, age, gender, preference information, and location information. Additionally, alternate videos are used in the next step of the user's preference procedure. Each category is subdivided according to specific conditions based on the user's information, whereas the mechanism illustrates subdivision in the second column of table (1) and classification based on subgrouping, which contains more detailed information. For example, the speed category in preference selection is further divided into jogging, fast running, and cycling [9, 12, 16, 17, 19].

The screening process of the fitness platform is shown in Figure 3, which highlights that the first half will complete the screening of clips in the video library according to the four categories of information. Apart from that, selected libraries use personal searching history to form effective fitness environment video recommendations. Moreover, this platform has a list of preferred videos based on types of user exercises. Especially for new users, the mentioned applications encourage them by presenting remarkable achievements. However, random fitness video suggestions can be carried out according to the initially selected video [10, 16].

Due to the short phase development time of the Chinese fitness platform, which tries to establish a set of physical assessments, individual physical exercise is just random and free movement without any restriction. At the present stage, the application is unable to rely on personal living standards or gender. The professional characteristics, physical fitness, and medical services are provided in a timely manner, which provides each athlete with specific guidance on the physical function to check health status.

## 3. Construction of Video-Based Collaborative Filtering Recommendation Model

### 3.1. Collaborative Filtering Algorithm

Collaborative filtering, as its name implies, consists of two parts: collaborative and filtering algorithms. The collaborative approach is a comprehensive judgment, which is based on the user's historical behavior records to provide assistance. Furthermore, the whole process helps them to make decisions. The end results of the filtering algorithm are the user's preference, while in the recommendation system, the collaborative filtering algorithm is utilized. This system is based on the similarity between the users to filter and complete the recommendation results. Different approaches are used for calculating the connection between users and items. Moreover, the collaborative filtering algorithm is further divided into the following three categories: user-based, item-based, and content-based [8, 16, 20].

The article "Internet-Based Approaches to Designing an Online Fitness Platform" was retracted in 2023. Reasons: unreliable results or conclusions; concerns about the data; concerns about the peer review; concerns about the citations.

#### 3.1.1. Content-Based Collaborative Filtering Recommendation Algorithm

This technique completes the entire process of recommendation through the content of items, as explained in Figure 4. Firstly, establish a recommendation list of similar items. For instance, during task A, two similar items from the libraries B and C are searched according to the size of similarity value. Secondly, determine the liking degree of the user of task A in order to accomplish the ranking of user A liking degree. Finally, the recommendation process is carried out for Item B and Item C of user A in combination with Item A [16].

### 3.2. Collaborative Filtering Recommendation Algorithm Based on Video

In this technique, the proposed videos are based on a filtering system. Effective implementation of videos for users proceeds through calculating the similarities between videos. In this case, the similarity concept is provided from users' search history and preferred exercise. Firstly, determine the similarity index between videos. Secondly, compare the history with the database to locate their preferences. The previous task of the consumer links the platform with the library to establish a list of certain videos. At the same time, the degree of relationship is further divided into size values. A higher value indicates a higher degree of likeness, which naturally ranks them higher in the endorsement list.

The similarity between two videos is calculated through the browsing history between users and endorsed videos, as shown in the following formula [2, 11, 12]:

(1) $$\begin{array}{c} w_{a,b}=\frac{\left|M\left(a\right)\cap M\left(b\right)\right|}{\sqrt{\left|M\left(a\right)\right|\left|M\left(b\right)\right|}}, \end{array}$$

where  *w*_*a*,*b*_ represents the resemblance between videos a and *b*. The molecular part in (1) represents the intersection of users who have watched video *a* and video *b*, which reflects their similarity. In the denominator, the product of the total number of people who have watched video *a* and the total number of people who have watched video *b* takes the square root operation. The final result represents the total number of watched videos. The ratio of similarity can be obtained by dividing the intersection value by the total number [4, 12, 18].

The article "Internet-Based Approaches to Designing an Online Fitness Platform" was retracted in 2023. Reasons: unreliable results or conclusions; concerns about the data; concerns about the peer review; concerns about the citations.

Normally obtained parameters in (1) are only the similarity between video, also not the probability of final user's viewing video. However, the similarity index needs to be multiplied by the user's interest in the original video. This mathematical approach leads to the most probable video, as shown in

(2) $$\begin{array}{c} P_{u,b}=\sum_{a\in N\left(u\right)\cap N\left(b,m\right)}w_{a,b}r_{u,a}, \end{array}$$

where  *P*_*u*,*b*_ represents the probability that user “*u*” likes video *b*, whereas “*a*” represents the video that user “*u*” has watched. *N*(*u*) represents the clips' set of all the types that user “*u*” likes to watch. *N*(*b*, *m*) represents the set of *m* video that is most similar to video “b.” This approach is used to find the recommendation list. Both videos are watched by user u, and one of the videos m is similar to video b. *w*_*a*,*b*_ has the same function as (1) in locating the adjacent contents between video *a* and video *b*, whereas *r*_*u*,*a*_ is probability value of users *u* interest in video “*a*” [15, 16, 21].

### 3.3. Popularity

This methodology work on three matching techniques: forward matching, reverse matching, and statistical matching. Finally, selection method is purely based on the word segmentation of user as given in Figure 5:

(3) $$\begin{array}{c} P\left(W|C\right)=\frac{P\left(W,C\right)}{P\left(C\right)}=\frac{P\left(W\right)P\left(C|W\right)}{P\left(C\right)}. \end{array}$$

However, it is inevitable to encounter the problem of popularity in video endorsement. For some current popular videos, the number of viewers will naturally arise, which leads to an inaccurate phenomenon in video simulation. Therefore, in order to improve the accuracy of recommendation results, it is essential to deal with the popularity problem between videos. Effectively punishing the popularity of video is used to be proceeded through decreasing the suggestion of that specific video. The punishment process for video popularity is shown in formula (3) [12].

(4) $$\begin{array}{c} w_{a,b}=\frac{\sum_{u\in M\left(a\right)\cap M\left(b\right)}1/\log\;1+\left|M\left(u\right)\right|}{\sqrt{\left|M\left(a\right)\right|\left|M\left(b\right)\right|}}. \end{array}$$

Comparing the video resemblance in (1) and (3) result in ∑_*u*∈*M*(*a*)∩*M*(*b*)_1/log  1+|*M*(*u*)|. User “*b*” who watched both video “*a*” and video “*b*,” a product factor 1/log  1+|*M*(*u*)|, should be added to in order to punish user “*u*.” Therefore, the influence of popular video on the data similarity calculation process needs to be limited.

The article "Internet-Based Approaches to Designing an Online Fitness Platform" was retracted in 2023. Reasons: unreliable results or conclusions; concerns about the data; concerns about the peer review; concerns about the citations.

Penalty factor before and after the enhancement of video popularity: the comparison results of recommendation in accuracy, recall rate, and coverage of the recommendation system are shown in Tables 2–4 collectively. The suggested result shows a slight improvement in accuracy, recall, and coverage. The popularity penalty factor occurs, which effectively improves the efficiency of the system which leads to the enrichment of the user's comfort level [12, 17].

Accuracy refers to the proportion where correct data (video) has a total number of recommendation results and its value lies between 0 and 1. Value close to 1 indicates that the accuracy factor is higher. The results are shown in Table 2.

However, recall rate refers to the proportion of the actual data in the final recommendation results. The similarity index value lies between 0 and 1. The value closer to 1 indicates a higher completeness probability [4, 21]. The results are shown in Table 3.

Coverage is an effective measure of the system's ability to exploit the long tail of videos. The process is expressed as the ratio of the recommended video, where the total number of videos is in the video library. The results are shown in Table 4.

The process of transforming the original data is known as feature extraction. Firstly, the raw data is converted into real vectors. There are many types of raw data such as numeric, discrete, text, images, and videos. Secondly, the model is generated after converting the original data into a real vector. For better understanding, the model is utilized to learn the hidden rules in the data. Furthermore, this model is achieved by transforming the features. Exploratory data analysis is performed for feature extraction [12].

The main framework features and functions included are as follows: HDFS widely used for the distribution of file systems; it is a file storage component of data application. MapReduce is a computing structure for distributed data. Hbase is a NoSql column family database, which supports billions of rows and millions of columns of data storage. Especially in critical circumstances, when data performance is time-sensitive, HDFS is used to execute the task. Hive uses hql for statistical analysis to generate query analysis [11]. This component is used to generate tasks performed on the MR by parsing hql. The typical application scenario is integration with Hbase. Kafka is distributed subscription-based messaging system, which is analogous to the function of the message queue. The data are reserved by self and then forwarded to the consumer for buffer adaptation. Flume is a system for massive log collection, aggregation, and transmission. Flume's main function is to collect and transmit data even it supports the data source input and output [11, 15].

The article "Internet-Based Approaches to Designing an Online Fitness Platform" was retracted in 2023. Reasons: unreliable results or conclusions; concerns about the data; concerns about the peer review; concerns about the citations.

### 3.4. Similarity Search Results

Partially parallel results of filtering algorithm based on videos, as shown in Figure 6, *x-* and *y-*axes, represent different video, respectively, whereas clustering results of similarity ranges from user A to user F are purely based on their search history. For example, users A, B, and C are close to each other in Figure 6, which depicts their relationship in terms of search history. When making video recommendations, these three users are linked and share common behaviors [1, 6, 16].

Generally, EDA technology is divided into two categories. The first type is visualization technology, including box plot, histogram, multivariate graph, chain graph, Pareto graph, scatter plot, stem, leaf map, parallel coordinates, yield ratio, scale analysis, target projection tracking, component analysis, multilinear analysis, nonlinear dimensionality, and reduction. The second type is the quantitative analysis based on mean, variance, quantile, kurtosis, and skewness.

Site intelligence has an effective wireless network environment. Sporting equipment is monitored through proper evaluation gadgets such as the treadmill by the smart running box. This sensing box includes data, points, online payment, and commercial services. Internet-based devices are connected with other personal accessories. Additionally, the user is in touch with the surroundings and keeps updates on upcoming sports and social events. Beside, fitness people communicate through the same platform. Consequently, the real-time interaction amongst them is improved. Communication between user and group assist in maintaining trust; thus, it ensures an optimal social experience [2, 8, 10].

### 3.5. The Mass Curve of Body

The user's body mass curve finally calculated by the system is shown in Figure 7, which includes four indicators: weight information, body fat rate, muscle rate, and BMI. Collected information regarding body mass is usually represented by a graph. The mass curve of the body is updated after 12 months. The mass curve of the body is shown in Figure 8.

This promotes the development of smart old-age industries. Consequently, it encourages web-based companies to cooperate with health organizations, which include cloud computing, big data, and health monitoring, and promote endowment smart terminal products. Additionally, old-age companies analyze in-service applications, community homes, and pensions. This method supports social welfare and supports institutions and communities over 85 years old to carry out “internet plus” health care services [2, 5, 19].

The article "Internet-Based Approaches to Designing an Online Fitness Platform" was retracted in 2023. Reasons: unreliable results or conclusions; concerns about the data; concerns about the peer review; concerns about the citations.

Moreover, this whole process promotes the development of security innovations and integration of basic information with social security by supporting the cards based on financial applications, pension, and medical transfer. Basically, the “Smart People Society Cloud” was created to improve the online business and interprovincial business system. Besides the above applications, it also assists in social insurance and online business operation [21].

Additionally, improvement in cultural digitalization takes place. Incorporate resources such as books and educational and nonlegacy information to boost the digitalization of heritage. Support cultural services, which include fairness, openness, and sharing. Encourage enterprises to carry out online shopping and offline experience. Apart from that, it develops new formats such as animation online games and artistic design. Generally, a public cloud platform is generated, which leads to the finalization of the digital industry. Consequently, online-based colorful park is programmed as “Internet +” innovation [15, 21].

The proposed structure stimulates a new model of an online health care system. The main theme is to promote medical services and mobile applications such as “Healthy Connect” and establish a service model of “Hospital +, Network Platform +, Pharmacy +, and Family+.” Public platform based on the “health cloud” for public health, medical services, and health management is organized on the basis of “one card.” Such alterations are implemented in hospitals and medical institutions to complete the issuance of health cards [10, 21].

Moreover, it encourages health campaigns through “Internet +” sports applications, fitness services, and communication. Consequently, health in the sports sector will improve, and the sports industry will develop. Other facilities are incorporated in constructing an “Internet +” platform to complete the design of national fitness [13, 21].

## 4. Conclusions

Internet-based platforms conveniently enhance the personalization of fitness information services and guidance. However, face-to-face interaction facilitates the public to achieve professional guidance on time. This integrated information directly assists users in accessing online gyms and sports venues through the Internet. Offline public participation in fitness and sports assisted professionals in forming a new model, National Fitness 2.0. This model includes an intelligent fitness system, sensing technology, and large storage to collect data. Additionally, it utilizes other technological approaches to obtaining frequency and user attributes. The active data content assists in achieving smart management. Challenges also come along, such as incomplete fitness facilities, gym closure, and other issues. By analyzing these existing problems, the proposed solutions try to promote the professional and intelligent development of national sports [2, 8, 9].

The article "Internet-Based Approaches to Designing an Online Fitness Platform" was retracted in 2023. Reasons: unreliable results or conclusions; concerns about the data; concerns about the peer review; concerns about the citations.

Feature transformation and feature learning are all data feature categories. The PCA and LDA methods of feature transformation can only deal with linear transformation, where the number of new features is limited by the number of input features. The feature learning adopts the deep learning method, which can extract more complex [1, 5].

The national fitness online platform based on mobile Internet mainly provides users with three services: correct learning of various fitness methods, recording of fitness activities, and recording of physical fitness. For the recommendation of fitness video, the collaborative filtering recommendation algorithm based on video is adopted in the platform, but the accuracy of recommendation still needs improvement. The classification of fitness videos can also be more accurate and professional. At the same time, family units can be added in the later stage of the platform, where the information feedback of each family user's physique can be watched so as to facilitate mutual care and mutual supervision.

## Figures and Tables

**Figure 1:** Framework of the online platform.

**Figure 2:** The type selection status of a citizen movement.

**Figure 3:** The process of video screening.

**Figure 4:** Content-based collaborative filtering recommendation algorithm.

**Figure 5:** The basic thought diagram of CCWS word segmentation.

**Figure 6:** Similarity graph based on a video.

**Figure 7:** Data system.

**Figure 8:** The mass curve of the body.

**Table 1:** Categories and category segmentation.

Categories	Category segmentation
Time	6.00–9.00, 9.00–12.00, 12.00–16.00 16.00–18.00, 18.00–22.00, and 22.00–6.00 (+1)
Age	7–12, 12–18, 18–24, 24–30 30–40, 40–50, 50–60, and 60+
Gender	Male Female
Types of activities	Walking pace running Yoga Tutorial lesson Fitness equipment Power equipment Ball
Location	Small indoor area Large indoor area Small outdoor area Large outdoor area Outdoor public fitness area

**Table 2:** The comparison of accuracy.

	Before joining the punishment (%)	After joining the punishment (%)
MovieLens 100k	33.48	33.48
MovieLens 1M	34.55	34.56
Videos	33.54	33.55

**Table 3:** The comparison of recall.

	Before joining the punishment (%)	After joining the punishment (%)
MovieLens 100k	14.59	15.01
MovieLens 1M	15.25	15.27
Videos	11.32	11.34

**Table 4:** The comparison of coverage.

	Before joining the punishment (%)	After joining the punishment (%)
MovieLens 100k	12.36	12.40
MovieLens 1M	14.07	14.11
Videos	18.73	19.81

The article "Internet-Based Approaches to Designing an Online Fitness Platform" was retracted in 2023. Reasons: unreliable results or conclusions; concerns about the data; concerns about the peer review; concerns about the citations.

## Data Availability

The data used to support the findings of this study are included within the article.
